RETRACTED

# Risk factor analysis combined with deep learning in the risk assessment of overseas investment of enterprises

**DOI:** 10.1371/journal.pone.0239635

**Published:** 2020-10-02

**Authors:** Xiuyan Xu

**Affiliations:** Accounting Institute, Xijing University, Xi’an, Shannxi, China; University College London, UNITED KINGDOM

## Abstract

To evaluate the overseas investment risks of enterprises and expand the application and development of deep learning methods in risk assessment, 15 national clusters are utilized as samples to analyze and discuss the overseas investment risk indicators of enterprises. First, based on the indicator system of overseas investment risks, five major types of investment risks are identified. Second, the Deep Neural Network (DNN) is introduced; a risk evaluation model is constructed for enterprise overseas investment. Finally, the investment attractiveness index in the Fraser risk assessment learning label is adopted as the evaluation results of the model. According to the classification of risks, the model is trained and its performance is tested. The results show that the major source of overseas investment risks includes basic resources, political systems, economic and financial development, and environmental protection. The corresponding risk score is high. North American country clusters and Oceanian country clusters have lower investment risks, while the investment risks in Africa, Latin America, and Asia are affected by multiple factors of the specific cities. This is closely related to the resources and legal systems possessed by the country clusters. This is of great significance for enterprises to conduct risk assessment in overseas investment.

## 1. Introduction

In the overseas investment activities of enterprises, risk is the most critical problem and challenge [1, 2]. Especially, for mining enterprises, their overseas investment projects are affected by multiple factors such as long periods and various uncertainties. The impact on the ecological environment is large. Under the action of multiple factors, there is a greater degree of uncertainty between the investment expenditure of mining enterprises and the expected benefits. Therefore, the application of scientific and effective solutions to assess the investment risks has great significance in reducing losses of enterprises and ensuring the utilization of overseas resources and energy. The assessment of investment risks has been extensively discussed by researchers. Wu et al. (2019) researched the risk management strategy of chemical industry clusters and found that when unexpected losses increased, enterprises were more inclined to adopt high-level investment strategies [3]. For the difficulty in calculating the weight of risk assessment indicators in traditional investment risk assessment models, Ren and Du (2018) constructed an industrial investment risk assessment indicator system from the levels of systemic risks and non-systematic risks; on this basis, they proposed a Support Vector Machine (SVM)-based industrial investment risk assessment model for the marine foreign trade and economic zone; the results suggested that the model could assess risks through empirical analysis [4]. Liu and Zeng (2017) adopted the system dynamics method to analyze and discuss the investment risks of renewable energy projects,' the results revealed that policy risks, technical risks, and market risks had greater impacts [5]. Yao et al. (2017) proposed a tactical exploration framework that applied grammar-based genetic planning to the generation and evolution of tactics in combat-level simulations, which could effectively reduce investment risks [6]. Due to its unique advantages, deep learning has been widely used in many fields [7]. The applications of deep learning methods in the field of risk or investment have been researched extensively. Xie et al. (2020) analyzed and discussed the application of deep learning in financial data processing, investment model, and investment strategy establishment, which had reference value for improving investors’ investment strategy and rate of return [8]. Sohangir et al. (2018) explored the application of Convolutional Neural Network (CNN) in stock market investment forecasting; they found that deep learning models could be effectively applied to financial analysis, and CNN had the best effect [9]. Liu (2019) believed that the prediction accuracy and portfolio optimization of financial risks were very important and compared the performance of Support Vector Machines (SVM) and Long Short Term Memory Recurrent Neural Networks (LSTM-RNNs) in classification; the results suggested that the latter had better performance, which was of great significance for maximizing investment profits [10]. Kim and Won (2018) proposed a new hybrid LSTM model and found that the model could be applied to the prediction of stock market volatility [11].

RETRACTED

The above research indicates that investment assessment and investment risks have been discussed a lot. At the same time, deep learning methods have been widely adopted in market forecasting and investment. Meanwhile, the assessment of overseas investment risks is less researched, let alone the applications of deep learning methods in overseas investment risk assessment.

The effective assessment of risks is influential. To build a risk assessment model for overseas investment of enterprises and evaluate investment risks scientifically and effectively, the Deep Neural Network (DNN) based on deep learning is introduced, which is an innovation. The built risk assessment model is built to provide a reference for enterprises to assess investment risks and reduce risks.

## 2. Method

### 2.1 Selection and construction of overseas investment risk indicator system

From the perspective of enterprises, overseas investment risks are affected by multiple factors, and the function of each influencing factor is very unclear. It is widely recognized that the overseas investment risks of enterprises are a huge and complex system. Therefore, it is necessary to design and construct an investment risk assessment system. During the entire process of constructing the assessment system, determining the construction principles and the composition of the investment risk influencing factors are the key links, which helps refining the influencing factors and indicators. On this basis, the review of literature, on-site inspections, and expert consultation are the means of model construction; in the meantime, the construction principles of scientificity, reliability, and comparability are persisted. The assessment system is divided into risk categories, project components, and risk factors. For the evaluation of venture capital, common methods include variance method [12], coefficient and capital asset pricing model [13], “A” scoring method [14], value-at-risk evaluation model [15], and comprehensive risk index model [16]. Due to the complexity of different country clusters, the comprehensive risk index evaluation method is adopted.

The risks in the overseas investment assessment system are divided into basic resources, economics and finance, political systems, environmental protection, and resources and energy. Then, these five categories are refined.

Under the category of basic resources, the investment goal is to improve the infrastructure equipment in the process of overseas investment and resource development of enterprises; specifically, it includes health care, basic communications, power energy, and land resources [17]. The category of economic and finance is correlated to the economic development and financial system in the destinations of overseas investment. The investment goal of this category is to promote the optimization of enterprise profits. The risk can be evaluated by the inflation rate and GDP. Here, this risk category is refined into economic growth, financing, changes in interest rates and exchange rates, inflation, credit systems, and total tax rates [18]. The risk category of political systems mainly characterizes the degree of political influences, as well as the stability of a particular country. This is a key factor in assessing the diplomatic situation, which also includes the level of rule of law and policy support. In particular, the major risk factors of the political system include regime alternation, contradictions and conflicts among surrounding powers, law system, social credit, foreign shareholding, and partners [19]. The risk factor category of environmental protection is essential for investment enterprises. When enterprises make overseas investments, they will always consider environmental protection factors, such as the legal requirements of environmental protection, the environmental law enforcement level of the investment destinations, and the impact of natural factors on environmental protection.

RETRACTED

Specifically, this category, a major risk factor, is refined into environmental law enforcement and environmental expenditures [20]. The risk factor category of resources and energy includes the development and utilization of minerals and other resources. Specifically, this category is refined into resource application potential and development conditions [21]. An overseas investment risk assessment system of enterprises including five major categories is thereby built. The details of categories are shown in Table 1 below.

**Table 1:** The composition of the risk assessment indicator system for overseas investment of enterprises.

Investment risk categories	Investment risk projects	Investment risk factors
Basic resources	Health care	A1 - Health care (+), risk (-)
	Basic communication	A2 - Infrastructure (+), risk (-)
		A3 - Communication conditions (+), risk (-)
	Resource and energy supply	A4 - Supply (+), risk (-)
Economic and finance	Economic situation	B1 - Economic growth (-), risk (+)
		B2 - Inflation (-), risk (-)
	Financial foreign exchange	B3 - Financing (+), risk (+)
		B4 - Interest rate and exchange rate changes (-), risk (-)
		B5 - Credit system (+), risk (-)
	Corporate taxes	B6 - Total tax rate (-), risk (-)
Political systems	Regime stability	C1 - Regime alternation (+), risk (-)
		C2 - Contradictions and conflicts among surrounding powers (+), risks (+)
	Legal governance	C3 - Law system (-), risk (-)
		C4 - Social credit (-), risk (-)
	Operating environment	C5 - Foreign shareholding (-), risk (-)
		C6 - Partners comply with the contract (+), risk (-)
Environmental protection	Environmental regulation	D1 - Law enforcement of environmental protection (-), risk (-)
		D2 - Environmental protection issue expenditure (-), risk (-)
Resources and energy	Resource conditions	E1 - Resource application potential (+), risk (-)
		E2 - Resource development (+), risk (-)

Note: “+” indicates greater degrees or greater risks, and “-” indicates smaller degrees or lower risks.

RETRACTED

### 2.2 Construction of investment risk assessment model based on deep learning network

Of late years, deep learning technology has developed rapidly. DNN has been applied in image recognition, text detection, and other fields. Compared with previous machine learning methods, deep learning technology has better performance in data fitting of complex factors [22, 23]. Therefore, the deep learning method is adopted to build the overseas investment risk assessment model of enterprises. The overall construction idea includes three steps: preliminary model construction, model training, and analysis and characterization of model performance. Deep learning technology includes a variety of models, for DNN, strong feature extraction ability, easy training, fast convergence speed, and simple structure composition are its characteristics [24]. Considering the characteristics of investment risk assessment, DNN is applied to the construction of the enterprise overseas investment risk assessment model.

In deep learning neural network models, the structure of DNN is different from traditional neural network models. It consists of the input layer, the hidden layer, and the output layer [25]. A basic model *Y*_*K*_ corresponding to DNN can be expressed as:

$$Y_{K}=f\left(\sum_{i=1}^{n}w_{iK}\times x_{i}+b_{K}\right)$$ (1)

In (1), *x*_*i*_ represents the neural unit node of the DNN, *w*_*iK*_ *b*_*K*_ represents the value of the weight, *b*_*K*_ represents the bias, and *Y*_*k*_ represents the activation function.

The training process of DNN is shown in Fig 1 below.

**Fig 1:** The training and testing processes of DNN.

On this basis, the input and output of DNN in overseas investment risk assessment are defined. *X* is utilized as the input value of the evaluation model, and the above five categories of investment risks are converted into corresponding risk indicators. First, the evaluation model is input into the sample feature dataset, which is represented by the following equation:

$$X=\left[\begin{array}{c} x_{1}\\ x_{2}\\ M\\ x_{L}\\ x_{L+1}\\ M\\ x_{L+U} \end{array}\right]=\left[\begin{array}{cccc} x_{1}^{1} & x_{1}^{2} & L & x_{1}^{F}\\ x_{2}^{1} & x_{2}^{2} & L & x_{2}^{F}\\ M & M & L & M\\ x_{L}^{1} & x_{L}^{2} & L & x_{L}^{F}\\ x_{L+1}^{1} & x_{L+1}^{2} & L & x_{L+1}^{F}\\ M & M & L & M\\ x_{L+U}^{1} & x_{L+U}^{2} & L & x_{L+U}^{F} \end{array}\right]$$ (2)

In (2), *F* represents the number of features corresponding to each data, which corresponds to the risk factor indicator in the assessment model; *L* represents the number of labeled data, which corresponds to the investment destination in the assessment model and the training sample; *U* represents the number of unlabeled data, which also corresponds to the test sample.

RETRACTED

If *Y* is the output value of the evaluation model, it will also correspond to the sample risk label dataset.

$$Y=\left[\begin{array}{c} y_{1}\\ y_{2}\\ M\\ y_{L} \end{array}\right]=\left[\begin{array}{cccc} y_{1}^{1} & y_{1}^{2} & L & y_{1}^{C}\\ y_{2}^{1} & y_{2}^{2} & L & y_{2}^{C}\\ M & M & K & M\\ y_{L}^{1} & y_{L}^{2} & L & y_{L}^{C} \end{array}\right]$$ (3)

In (3), *C* represents the number of categories corresponding to the sample label. Refined into the investment risk assessment, the investment risks are divided into five different levels; level I indicates that no investment can be made, level II indicates that the investment risk is serious, level III indicates that the investment risk is high, level IV indicates that the investment risk is average, and level V indicates that the investment risk is low. These five different risk levels correspond to five label categories and the realization of the labeling rules, which can be expressed as:

$$y_{j}^{i}=\{\begin{array}{cc} 1-20 & x_{j}\in I\\ 21-40 & x_{j}\in II\\ 41-60 & x_{j}\in III\\ 61-80 & x_{j}\in IV\\ 81-100 & x_{j}\in V \end{array}$$ (4)

For the sample dataset in the input investment risk assessment model, feedforward calculation should be utilized to judge and express the input data features. After successive propagation throughout the layers, the data dimensionality is finally reduced. In this process, the corresponding data are constantly becoming abstract, and finally, the result can be predicted. The risk assessment model of enterprise overseas investment built here is actually a process of reducing multidimensional data to five dimensions. To solve this problem, the feedforward propagation of information in DNN can be expressed as:

$$Z^{\left(p\right)}=W^{\left(p\right)}\cdot f_{p}\left(Z^{\left(p-1\right)}\right)+b^{\left(p\right)}$$ (5)

In (5), *Z*^(*p*)^ represents the specific state of the eigenvalues corresponding to the *p*-tier investment risk assessment, *W*^(*p*)^ represents the weight matrix, *f*_*p*_ represents the activation function corresponding to the eigenvalues of the *p*-tier investment risk assessment, and *b*^(*p*)^ is the offset.

The information is passed successively throughout the layers in DNN, and finally, the output of the network can be obtained. Considering that data can have limitations in the target countries or regions for enterprises investment overseas, the application of labeled data can play an important role in the training of the network. If there is a set of data samples (*x*^(*i*)^, *y*^(*i*)^):

The corresponding output of the neural network after the feedforward propagation is *f*(*x*|*w*,*b*):

Then, the corresponding objective function *O*(•) can be expressed as:

$$O\left(W,b\right)=\sum_{i=1}^{N}O\left(W,b;x^{\left(i\right)},y^{\left(i\right)}\right)+\frac{1}{2}\lambda ∥W{∥}_{F}^{2}$$ (6)

In (8), *W* represents the weight matrix corresponding to each layer, and *b* represents the bias vector corresponding to each layer in the neural network. Based on the goal of minimizing investment risk output, the gradient descent method is applied to realize the iteration and update of parameters. The corresponding calculation is:

$$W^{\left(p\right)}=W^{\left(p\right)}-\delta \sum_{i=1}^{N}\left(\frac{\partial O\left(W,b;x^{\left(i\right)},y^{\left(i\right)}\right)}{\partial W^{\left(P\right)}}\right)-\lambda W$$ (7)

In (9), *δ* represents the update rate corresponding to the parameter, and *λ* represents the parameter. Furthermore, the error term is defined as:

$$e^{\left(p\right)}=f_{p}^{\prime }\left(Z^{\left(P\right)}\right)⊙{\left(W^{\left(p+1\right)}\right)}^{T}\cdot e^{\left(p+1\right)}$$ (8)

In (10), ⊙ represents the dot product operator of vectors.

RETRACTED

After obtaining the error term corresponding to each layer, the gradient value corresponding to each layer parameter can be obtained.

According to above analysis, the entire training process of DNN is achieved through the calculation of the state and activation value of each layer, as well as the calculation of the error corresponding to each layer in the neural network, which helps update the relevant parameters.

The expression level of DNN also plays an extremely important role, which can be achieved by the introduction of nonlinear activation functions. The logistic function, tanh function, and ReLU function are the most commonly used activation functions in traditional neural network models. However, the first two activation functions have the problem of gradient disappearance during neural network training [26]. Therefore, in the proposed model, ReLU is used as the activation function, and its corresponding equation is:

$$f\left(x\right)=\max\left(0,x\right)=\{\begin{array}{cc} 0, & x\leq 0\\ x, & x>0 \end{array}$$ (9)

Compared with the other two activation functions, the gradient calculation corresponding to the ReLU function can be expressed as:

$$f\left(x\right)=\{\begin{array}{cc} 1, & x>0\\ 0, & x<0 \end{array}$$ (10)

This makes the problem of gradient disappearance in the entire backpropagation process alleviated.

### 2.3 Training and testing of the risk assessment model for enterprise overseas investment

To test the effectiveness of the DNN-based enterprise overseas investment risk assessment model, the Fraser risk assessment is chosen as the learning label. This risk assessment includes multiple countries and regions [27, 28]. Here, countries and regions that have continuity in the Fraser risk assessment learning label from 2018 to 2019 are selected as the research samples. Specifically, a total of 15 countries are included as the target countries. Besides, President Xi Jinping of China has visited all the included countries, sharing close cooperative relations with China. In addition, the selected countries have rich resources such as minerals. The five risk assessment levels proposed above are utilized to analyze and characterize the proposed DNN-based enterprise overseas investment risk assessment model. The selected research samples are shown in Table 2 below.

RETRACTED

**Table 2:** Selection of research samples.

Regions	Sample countries	Regions	Sample countries
Asia	Indonesia	Africa	Congo
	India		Zambia
	Philippines		South Africa
Europe	Finland	Latin America	Peru
	Sweden		Brazil
			Chile
North America	The United States		
	Canada		Argentina
Oceania	Australia		

Specifically, the final selected sample set is the investment risk characteristic data corresponding to 15 countries from 2018 to 2019, including a total of 165 research samples containing 5710 characteristic values. Among them, the selected training samples include a total of 124 research samples containing 4284 feature values; the selected test samples include a total of 41 research samples containing 1426 feature values. The evaluation indicators of this enterprise overseas investment risk assessment model are shown in Table 1 above. Furthermore, for output *Y* of the risk assessment model, the investment attractiveness index of the target country or region in the Fraser risk evaluation learning label is adopted as the evaluation result of the model. In addition, the corresponding label of the model output is divided into five risk levels according to the corresponding scores. Therefore, the model is trained and its performance is tested.

## 3. Results

### 3.1 Analysis of the risk assessment indicators for enterprise overseas investment in American country clusters

During 2018–2019, the selected overseas investment risk assessment indicators for North American country clusters and Latin American country clusters are shown in Fig 2A–2D below.

**Fig 2:** The results of the overseas investment risk assessment of North America and Latin America country clusters in 2018–2019. (a) Risk categories of basic resources and economic and finance in 2018; (b) Risk categories of political system, environmental protection, and resources and energy in 2018; (c) Risk categories of basic resources and economic and finance in 2019; (d) Risk categories of political system, environmental protection, and resources and energy in 2019.

RETRACTED

Data analysis shows that the risk assessment indicators of the two countries in North America, the United States and Canada, show different indicators among the five risk levels. However, because the United States and Canada have richer reserves of resources and energy, coupled with a higher level of economic development, better political systems, and sound infrastructure, the overall investment environment is better, and the overall investment risks are also lower. In contrast, however, several countries in Latin America have different levels of investment risks. This is mainly due to differences in the level of economic development between countries, as well as the differences in the supply of basic resources and the rule of law system.

### 3.2 Analysis of the risk assessment indicators for enterprise overseas investment in Asian country clusters

During 2018–2019, the selected overseas investment risk assessment indicators for Asian country clusters are shown in Fig 3A–3B below.

**Fig 3:** The results of the overseas investment risk assessment of Asian country clusters in 2018–2019. (a) Risk categories of basic resources and economic and finance; (b) Risk categories of political systems, environmental protection, and resources and energy.

Data analysis shows that Asian countries have richer resources and energy reserves. However, due to multiple factors, such as the development level of industries, professional skills, and capital supply, generally, these countries show higher investment risks. This is inseparable from a country’s political development trends and geographic location.

### 3.3 Analysis of the risk assessment indicators for enterprise overseas investment in African country clusters

During 2018–2019, the selected overseas investment risk assessment indicators for African country clusters are shown in Fig 4A–4B below.

**Fig 4:** The results of the overseas investment risk assessment of African country clusters in 2018–2019. (a) Risk categories of basic resources and economic and finance; (b) Risk categories of political systems, environmental protection, and resources and energy.

Analyzing the risk assessment indicators of each risk level shows that African country clusters also have abundant resources and energy reserves. However, because the overall level of economic development is poor, these countries are highly dependent on mineral resources and energy exports. In addition, the political system are often traditional so that the degree of implementation is also poor. The political situation in Africa is generally stable but partially turbulent, leading to a higher level of investment risk.

RETRACTED

### 3.4 Analysis of the risk assessment indicators for enterprise overseas investment in European and Oceanian country clusters

During 2018–2019, the selected overseas investment risk assessment indicators for European and Oceanian country clusters are shown in Fig 5A–5B below.

**Fig 5:** The results of the overseas investment risk assessment of European and Oceanian country clusters in 2018–2019. (a) Risk categories of basic resources and economic and finance; (b) Risk categories of political systems, environmental protection, and resources and energy.

Changes in the risk indicators show that the overall resource and energy reserves of the European country clusters are general; however, the basic resources, such as infrastructure, are sound and complete. The overall macroeconomic development level is lower. The overall risks at all levels are lower in several cities. Australia, a representative country of Oceania, has abundant minerals, coal, and other natural resources, with independent legislation among states, stable political trends, and sound infrastructure; therefore, the overall investment environment is good.

## 4. Discussion

The above analysis suggests that a country’s infrastructure, health care conditions, economic development level, environmental protection conditions, and political system are the key components that affect its risks of enterprise overseas investment [29, 30]. In contrast, North American countries are more favorable target countries for overseas investment, which are inseparable from their resources and energy, health care conditions, economic development, and political systems. Among the investment risks, the biggest disadvantage of the North American clusters is that if the investment is associated with mining, due to the high requirements for environmental protection, the labor factors and other issues must be considered. Meanwhile, in Latin American clusters, the main problems are the level of economic development and the imperfections of infrastructure and legal construction. In the meantime, considering the actual situation during the current COVID-19 (Corona Virus Disease 2019) pandemic, the situations in the United States and other countries are severe, which also needs to be noted in investment. Asian countries have abundant resources and energy reserves; besides, the overall political development situation is stable [31]. However, the policies for investment are not perfect and stable enough. Changes in leadership will trigger adjustments and changes in policies; therefore, problems in the efficiency and concepts of the government have led to an increase in investment risks. In the meantime, the presentation of the final result of investment risks is inseparable from a country’s geographic location.

RETRACTED

In terms of development stage, Africa is still in the initial period of industrialization. Although the momentum of development in recent years has become stronger, the overall facilities and systems need to be improved. In addition, the health care conditions in Africa are backward. Natural disasters and infectious diseases occur frequently. This is a concrete manifestation of the risks of African country clusters in overseas investment, which is also an aspect that needs attention. The enterprise overseas investment risks of European and Oceanian clusters also illustrate the important role of several risk factors in investment.

## 5. Conclusion

A total of 15 country clusters with different geographical locations are chosen as the research objects. Based on risk factor analysis, the DNN-based enterprise overseas investment risk assessment model is tested. The results suggest that the investment risk indicators can clearly show the level of investment risks. The investment risk level of each country is comprehensively affected by basic resources and energy, political systems, and economic and financial development levels. The above results have provided basic data support for the risk assessment of enterprises overseas investment. However, the assessment of enterprise investment risks is still in the exploratory stage. Affected by multiple objective factors, the sample data only include the risk indicators during 2018–2019. As the research continues to be expanded, the sample data will be increased in the future to obtain more valuable results.

## Supporting information

S1 Data (RAR)
